The article "Predicting the Physician's Specialty Using a Medical Prescription Database" was published in 2022. Journal: Comput Math Methods Med.

# Predicting the Physician's Specialty Using a Medical Prescription Database

**DOI:** 10.1155/2022/5871408

**Published:** 2022-09-16

**Authors:** Mahboube Akhlaghi, Hamed Tabesh, Behzad Mahaki, Mohammad-Reza Malekpour, Erfan Ghasemi, Marjan Mansourian

**Affiliations:** ^1^Department of Biostatistics and Epidemiology, School of Health, and Student Research Committee, School of Health, Isfahan University of Medical Sciences, Isfahan, Iran; ^2^Department of Medical Informatics, School of Medicine, Mashhad University of Medical Sciences, Mashhad, Iran; ^3^Department of Biostatistics, School of Health, Kermanshah University of Medical Sciences, Kermanshah, Iran; ^4^Non-Communicable Diseases Research Center, Endocrinology and Metabolism Population Sciences Institute, Tehran University of Medical Sciences, Tehran, Iran; ^5^Epidemiology and Biostatistics Department, School of Health, Isfahan University of Medical Sciences, Isfahan, Iran

## Abstract

**Purpose:**

The present study is aimed at predicting the physician's specialty based on the most frequent two medications prescribed simultaneously. The results of this study could be utilized in the imputation of the missing data in similar databases. *Patients and Methods*. The research is done through the KAy-means for MIxed LArge datasets (KAMILA) clustering and random forest (RF) model. The data used in the study were retrieved from outpatients' prescriptions in the second populous province of Iran (Khorasan Razavi) from April 2015 to March 2017.

**Results:**

The main findings of the study represent the importance of each combination in predicting the specialty. The final results showed that the combination of amoxicillin-metronidazole has the highest importance in making an accurate prediction. The findings are provided in a user-friendly R-shiny web application, which can be applied to any medical prescription database.

**Conclusion:**

Nowadays, a huge amount of data is produced in the field of medical prescriptions, which a significant section of that is missing in the specialty. Thus, imputing the missing variables can lead to valuable results for planning a medication with higher quality, improving healthcare quality, and decreasing expenses.

## 1. Introduction

Population aging, urbanization, and consequently noncommunicable disease (NCD) prevalence have led to the escalation of medication consumption per capita globally [1]. According to the United Nations Office on Drugs and Crime (UNODC) report in 2018, about 80% of the population between the ages of 15 and 64 in Asia are taking medications [2]. Considering the prevalence of NCDs and their associated prescribed healthcare services, insurance claimed data, even in a short period, provides an invaluable source of big data.

Heterogeneity is one of the big data characteristics, which leads to obtaining biased or even erroneous results [3, 4]. Although clustering on big data to create homogeneous clusters is an essential step for the subsequent analyses [5], it also produces intermediary results that researchers could use to interpret the relation of variables within clusters [6, 7]. In addition, missing data may affect the valence of the data in big data applications [8]. Therefore, imputing missing data leads to reasonable, valuable, and unbiased results. Among numerous studies that investigated medical prescriptions in various ways [9–11], a considerable proportion reported a significant rate of up to one-third for the physician's specialty missingness [12–17]. Despite the provision of a remarkable increase in the accuracy of disease labeling of patients, one of the overlooked applications of studying prescriptions is predicting the physician's specialty.

To the best of our knowledge, limited studies have been conducted to predict the specialty of physicians using machine learning methods on big data. The present study is aimed at predicting the physician's specialty based on the most frequent two medications prescribed simultaneously. The results of this study could be utilized in the imputation of the missing data in similar databases.

## 2. Materials and Methods

### 2.1. Data Source

The data used in the study had been registered in the second populous province of Iran (Khorasan Razavi) from April 2015 to March 2017. The data included the fields of prescription ID, patient ID, medication, and prescription date, as well as physician's specialty, gender, and age. Also, each record of the data represents a single medication of prescription.

### 2.2. Data Manipulation and Analysis

An essential step at the beginning of the analysis process is data wrangling. In this study, data was retrieved from 4 SQL tables and preprocessed via R language. As the variables in this step contained both quantitative and qualitative measures, KAy-means for MIxed LArge datasets (KAMILA) clustering was implemented, which is suitable for clustering mixed-type data [18]. In this step, the variables included in the clustering were age of physician, medication, insurance company, prescription month, sex of physician, physician specialty, corticosteroid, and antibiotic. Moreover, specialties with ages between 22 and 85 years old are included in the study. Also, prescriptions with only one medication were excluded from further analysis. Based on the expert opinion, the number of clusters has been determined to be four.

After evaluating the results of the first step, all combinations of two medications (2-combs) in every prescription were derived, and a new data set was developed.

In similar studies which investigated disease prediction, the random forest (RF) model was suggested as the superior model with the highest performance compared to other well-known predictive models such as support vector machine (SVM), Naïve Bayes algorithm, and logistic regression [19–22]. Furthermore, RF is convenient in situations including more than two classes [23]. When specialties are missed in a database, there is no information available about specialist characteristics. So, the study has proposed an RF model that uses characteristic-free variables as predictors, i.e., 2-combs.

At last, in order to predict the specialty based on prescription patterns, the following actions have been done.

The RF method has been fitted as the following phases:

- The count of the 2-combs was calculated and sorted in a descending order
- For each specialty, the selected proportions of the prescribed 2-combs were calculated
- Data were restructured as wide format
- To select the appropriate variables as predictors in the RF model, several RF models were fitted on the data using the first *n* most frequent 2-combs (*n* = 1, 2, ⋯, 40)
- Selecting variables to achieve appropriate accuracy
- Checking the validation of the model using the accuracy index

In this approach, the first 25 most frequent combinations have been used as variables, and the physician's specialty was considered the response. The 7354 specialties have been split into training and validation datasets by a 70/30 proportion. Therefore, 5160 and 2194 observations were randomly allocated to training and test subsets, respectively.

To carry out the research aim, R 4.1.2 programming language has been used to develop codes, and the RStudio environment was applied to implement and execute them. As well, Apache Spark framework 3.1.0 via “sparklyr” R library along with “tidyverse” and “vroom” libraries was used for data wrangling. Besides, other libraries like “kamila” and “RandomForest” were used for analyses. Finally, “ggplot2” and “ggtext” have been applied to make visualization. A configured computer with 64 GB of RAM and a 32-core Intel CPU was used.

## 3. Results

The study results were obtained from 17,137,949 prescriptions prescribed by 30,544 physicians. 18,620 (61%) were related to male practitioners. The means of physician's age were 51.9 and 42.1 for males and females, respectively. In addition, general practitioners (GPs) constituted 20,081 (65.7%) of total physicians.

In the first step, KAMILA clustering was performed on prescription records.  Figure 1 provides overall sight of the distribution of each specialty in four clusters. For example, endocrinology and nephrology were concentrated in cluster 1.

As shown in Figure 2, the high-prescribed antibiotics (i.e., ciprofloxacin, azithromycin, cephalexin, chloramphenicol, and doxycycline) were concentrated in cluster 2. Results represented that GPs have prescribed the majority of the antibiotics. In addition, ibuprofen and diclofenac, two well-known nonsteroidal anti-inflammatory drugs (NSAIDs), were primarily categorized in clusters 1 and 4, respectively. Furthermore, dexamethasone was mainly categorized in clusters 3 and 4.

Variations and overlaps of medicines across specialty levels became a motivation factor in evaluating the 2-combs in another way. So, Figure 3 represents the five highest frequent 2-combs in each specialty.

The results of the RF classification model are presented as follows.

According to Figure 4, the value of accuracy in the 25th 2-combs tended to be a constant. The final RF model was fitted using the 25 most frequent 2-combs, which has the optimal accuracy of 0.74 in the validation dataset.

Figure 5 presents the mean decreased accuracy by deleting each predictor of the model, and it also represents each predictor's importance. So, the combination of amoxicillin and metronidazole between the 25 first combinations contributed the most to accuracy. Also, the combination of ASA and atorvastatin in Figure 3 appeared in several specialties as the most frequent 2-combs have the fourth accuracy rank in Figure 5. To predict the specialty, the findings of the study can be applied to any similar medical prescription database, which is provided in a user-friendly R-shiny web application (https://mahboube-akhlaghi.shinyapps.io/SpecialtyPrediction).

## 4. Discussion

The present study focused on predicting specialty based on the RF model on 17,265,238 prescriptions. Also, the method of this study is in line with numerous previous studies which have focused on disease prediction [19, 24]. Many studies presented the RF model's superiority over some machine learning methods [19].

Shirazi et al. used a community detection algorithm to identify the real specialty of physicians in prescription databases [25], which was a subjective method. In the present study, the authors tried to predict missing specialties differently. In the study, the 2-combs were utilized to predict the physician's specialty using the RF model.

However, the main findings of the study showed that the RF method could precisely predict the physician's specialty using the proportion of their most frequent 2-comb prescriptions. In addition, knowledge about the patterns of the prescription data can help better treatment and investigate the side effects of 2-combs. In this case, the combination of amoxicillin-metronidazole has the 21st rank among the 25 most frequently selected variables, which has the highest importance in making an accurate prediction. This is despite the fact that the recent systematic review and meta-analysis research about simultaneously amoxicillin/metronidazole usage in periodontitis treatment has shown positive short-term effects [26]. In addition, considering the extracted results showed that acetaminophen existed in several 2-combs. Several studies presented evidence that acetaminophen has adverse effects on certain human organs (for example, the liver) [27–29]. Moreover, some recent studies have presented simultaneously prescribing ASA and atorvastatin. He et al.'s research demonstrated the strong effect of ASA and atorvastatin 2-combs on inhibiting the growth of prostate cancer cells [30]. Other studies provided evidence of the merit of using these 2-combs in preventing and treating cardiovascular disease and severe sepsis [31–34]. Also, in many 2-combs, one of the medications was antibiotics. However, adverse events and antibiotic resistance are a well-acknowledged global problem [35, 36].

Finally, we found that general practitioners had the most outpatients. One reason for it is family physicians' issues [37]. Also, the services of general practitioners have a less economic burden on the patients than specialty physicians' services. Further, the prescribed medications were more related to the diseases such as colds and allergies, which patients often refer to a general practitioner. The observations in this study are limited to the insurance claimed database registry. However, in Iran, many prescriptions do not cover by insurance companies, and this issue is a specific limitation of the study.

## 5. Conclusion

In the study, we predict the physician's specialty by using the proportion of their most frequent 2-comb prescriptions. Today, a huge amount of data is produced in the field of medical prescriptions, which a significant section of that is missing in the specialty [12–17]. So, imputing the missing can lead to valuable results for planning a medication with higher quality, improving healthcare quality, and decreasing expenses [38–40].

## Figures and Tables

**Figure 1:** The heatmap plot of the specialty variable in four clusters.

**Figure 2:** The five highest frequent medications for each specialty in four clusters.

**Figure 3:** The five highest frequent 2-combs in each specialty.

**Figure 4:** The accuracy of the RF models against the number of most frequent 2-combs used as predictors.

**Figure 5:** The mean decreased accuracy by deleting each predictor of the model.

## Data Availability

The raw data used to support the findings of this study are restricted in order to protect patient privacy, but the aggregated data are available from the first author upon request.

## Abbreviations

NCDs: Noncommunicable diseases
UNODC: The United Nations Office on Drugs and Crime
KAMILA: KAy-means for MIxed LArge datasets clustering
RF: Random forest
SVM: Support vector machine
GPs: General practitioners
NSAIDs: Nonsteroidal anti-inflammatory drugs.
